# Grey Relational Analysis of Lower Limb Muscle Fatigue and Pedalling Performance Decline of Elite Athletes during a 30-Second All-Out Sprint Cycling Exercise

**DOI:** 10.1155/2021/6755767

**Published:** 2021-12-13

**Authors:** Lejun Wang, Hua Yang, Guoqiang Ma, Mingxin Gong, Wenxin Niu, Tianfeng Lu

**Affiliations:** ^1^Sport and Health Research CenterPhysical Education Department, Tongji University, Shanghai, China; ^2^Shanghai Research Institute of Sports Science, Shanghai 200030, China; ^3^Shanghai Yangzhi Rehabilitation Hospital, Tongji University School of Medicine, Shanghai 201619, China

## Abstract

The 30-second all-out sprint cycling exercise is a classical sport capacity evaluation method, which may cause severe lower limb muscle fatigue. However, the relationship between lower limb muscle fatigue and the decline in exercise performance during 30-second sprint cycling remains unclear. In this study, ten cyclists volunteered to participate in a 30-second all-out sprint cycling while power, cadence, and surface electromyographic (EMG) signals of eight lower limb muscles were recorded during the exercise. EMG mean frequency (MNF) of each lower limb muscle group was computed for every 3-second epoch based on wavelet packet transformation. Grey relational grades between pedalling performance and the EMG MNF of each lower limb muscle group during the whole process were calculated. The results demonstrated that EMG MNF of the rectus femoris (RF), vastus (VAS), gastrocnemius (GAS), and tibialis anterior (TA) progressively tired during a 30-second all-out sprint cycling exercise. Of the muscles evaluated, the degree of fatigue of TA showed the greatest association with exercise performance decline, whereas the muscle fatigue of RF, VAS, and GAS also significantly impacted exercise performance during a 30-second all-out sprint cycling exercise.

## 1. Introduction

The 30-second all-out sprint cycling exercise is a commonly used method in evaluating the anaerobic endurance capacity of lower limb muscles and has been widely adopted in sports training for cyclists [1]. As a vigorous exercise, 30-second all-out cycling causes severe lower limb muscle fatigue, which manifests as a decline in exercise performance [2, 3]. In fact, muscle fatigue occurs as early as five seconds in this intensive exercise [1, 4]. As the decline in exercise performance during 30-second sprint cycling is mainly determined by the fatigue of lower limb muscles, investigating the relationship between lower limb muscle fatigue and changes in exercise performance may further help in understanding the movement and aid training programme design.

Previous research evaluating muscle fatigue has mainly focused on total muscle fatigue at the end of the exercise or fatigue development in only a few muscles [2, 4]. Furthermore, earlier studies did not simultaneously quantify the development and progression of muscle fatigue in multiple lower limb muscles during 30-second sprint cycling. As different muscles have different functional roles during pedalling exercise, the process of fatigue development of each lower limb muscle can differ significantly [3, 5]. For example, muscle activity of the quadriceps decreased by approximately 8% during 30-second sprint cycling, whereas that of the gastrocnemius (GAS) decreased by up to 15%, indicating an unbalanced development of fatigue for the two muscle groups [5–7]. Thus, the relationship between the fatigue development of each lower limb muscle and changes in exercise performance during 30-second sprint cycling remains unclear.

Previous research has commonly evaluated local muscle fatigue using surface electromyography (EMG) signal processing. The efforts of several studies have yielded signal-based quantitative criteria of fatigue in both static and dynamic motor tasks [8–10]. Among comparisons of the utility of different methods to evaluate muscle fatigue, the wavelet transform has better accuracy and precision than those obtained from other time-frequency analysis methods in processing nonstationary EMG signals recorded during dynamic contractions [11]. In particular, Wang et al. [4] found that the grey relational grade between the mean frequency (MNF) derived from the wavelet transform of EMG and pedalling performance was as high as 0.78. Based on this finding, MNF exhibits superior utility to other indices in muscle fatigue evaluation induced by sprint cycling exercise, suggesting that the fatigue of lower limb muscles during a 30-second all-out cycling exercise can be assessed well using the MNF of EMG signals. Moreover, grey relational analysis is a crucial method to reflect the uncertainty in grey system theory, which was first initiated by Deng [12]. As the approach is appropriate for solving complicated interrelationships among multiple factors and variables, it may provide insights for exploring the relationship between exercise performance and fatigue development of lower limb muscles during 30-second all-out sprint cycling [13, 14].

This study determined the impact and contribution of fatigue from each lower limb muscle (or muscle group) to the exercise performance decline during a 30-second all-out cycling exercise by evaluating the grey relational grade between the degree of muscle fatigue and the decline in exercise performance. The extent of fatigue of each muscle was quantified by the MNF derived from wavelet packet transformation of EMG, whereas exercise performance decline was estimated by decreased rates of power output and cadence.

## 2. Materials and Methods

### 2.1. Participants

The sample size was estimated prospectively using G*∗*power v3.1.0 (Franz Faul, University of Kiel, Germany) with a level of 0.05 and a power of 0.95. We used a conservative effect size of 0.6 based on a previous study [15]. As a result, the sample size was estimated to be eight subjects. To allow for study withdrawal and dropout, we decided to recruit an additional two participants. Thus, the planned sample size of this study was 10.

On this basis, seven male and three female cyclists, with a mean age of 21.5 ± 4.67 years, a height of 175.0 ± 8.3 cm, a weight of 75.4 ± 10.91 kg, and a BMI of 24.50 ± 1.83, were recruited from the Shanghai Professional Cycling Team to participate in the study. The cyclists trained 6 days a week for 8 hours a day for more than 7 years and competed in Chinese national track cycling events. None of the cyclists received ergogenic aids or performance-enhancing drugs. Participants refrained from strenuous physical activity 24 h before the experiment and were screened using a questionnaire to ensure that they had not suffered a lower-body injury or other health issues that may affect performance. The experimental design was approved by the Ethics Committee of Tongji University.

### 2.2. Experimental Protocol

The experiment was conducted in a laboratory with an indoor temperature maintained at approximately 24°C and comprised a warm-up exercise and a test exercise (Figure 1). All exercises were performed on a Wattbike Pro air-braked ergometer (Wattbike Ltd., Nottingham, UK). After familiarisation with the laboratory equipment and test protocol, participants undertook a continuous warm-up on an air-braked ergometer for 5 min. The resistance was set at level 3 and the cadence at 90 rpm. Following a 3 min rest period, participants then completed a 30-second all-out sprint cycling. During the test, the saddle height and position of the participant on the ergometer were adjusted according to the setup of the cyclist's own bike, and the crank length was 170 mm for the experiment. Participants maintained a consistent bent posture with the hip fixed to the saddle and feet fixed to the pedals via straps during the pedalling exercise [16].

The air resistance on the Wattbike ergometer, which allowed a setting between 1 and 10, was set corresponding to the maximum power output that the participant produced during the all-out cycling exercise. According to the Wattbike technical documentation of the manufacturer, air resistance settings at levels 6 and 10 on the Wattbike ergometer result in a power output of 45 and 55 W at a cadence of 40 rpm, respectively, and 785 and 1045 W at a cadence of 130 rpm, respectively. Therefore, in this study, the ergometer was set to an air resistance level of between 8 and 10 for male cyclists and between 6 and 8 for female cyclists. Verbal encouragement was given to all participants to promote maximal engagement. In addition to the EMG signal acquisition, performance data (power and cadence) were recorded from the bike pedals at a sampling rate of 1 Hz. Surface EMG signals and Wattbike data were synchronised using a trigger that starts the EMG and Wattbike data sampling software simultaneously.

The air resistance on the Wattbike ergometer, which can be set between 1 and 10 levels, was set to correspond to the maximum output power that the participant can produce during the all-out cycling exercise. According to the Wattbike technical documentation, levels 6 and 10 of air resistance on the Wattbike ergometer result in power *s* of 45 and 55 W at a cadence of 40 rpm and 785 and 1045 W at a cadence of 130 rpm. As a result, in this study, the ergometer was set to level 8∼10 for seven male cyclists and level 6∼8 for three female cyclists. Verbal encouragement was given to all participants to promote maximal engagement. Along with the EMG signals, the performance data (power and cadence) were recorded from the bike pedals at a sampling rate of 1 Hz. Surface EMG signals and Wattbike data were synchronised by a trigger which can start the EMG and Wattbike data sampling software simultaneously.

### 2.3. EMG Measurement

Eight muscles of the right lower limb were selected for surface EMG measurement, namely, rectus femoris (RF), vastus lateralis (VL), vastus medialis (VM), biceps femoris (BF), semitendinosus (ST), tibialis anterior (TA), gastrocnemius lateralis (GAS), and soleus (SOL). Following the recommendations of the Surface ElectroMyoGraphy for the Noninvasive Assessment of Muscles (SENIAM) project [17], the skin of the electrode sites was identified, shaved, lightly rubbed, and cleaned using alcohol swabs to reduce impedance before EMG measurement. Surface EMG signals were recorded using a ME 6000 P8 Surface EMG acquisition instrument (Mega Electronics System, Kuopio, Finland) with bipolar Ag/AgCl electrodes with a 2 cm interelectrode distance. The sampling frequency of EMG signals was 1000 Hz. The electromyogram electrode locations of RF, VL, VM, BF, ST, TA, GAS, and SOL are shown in Figure 2.

### 2.4. EMG, Power, and Cadence Data Processing

Firstly, raw EMG signals were bandpass filtered at 5–500 Hz offline using a 4^th^ order zero-phase-shift Butterworth filter. Next, the EMG signal of each muscle was segmented for each 3-second epoch with no overlap, and the MNF based on wavelet packet transformation was calculated for each EMG segment. The values of muscles with the same function were combined and averaged (e.g., VL and VM were combined into VAS, BF and ST were combined into HAM). Correspondingly, power and cadence were averaged for every 3-second epoch for each participant during the intensive all-out cycling exercise. Since each participant was not fatigued in the first period, data of the 2^nd^ to 10^th^ periods of the 30-second all-out cycling exercise were used for the analysis.

In the wavelet packet transform analysis of surface EMG signals, the Daubechies (db6) wavelet was implemented for wavelet packet decomposition and reconstruction, and the MNF was calculated on this basis, using the following formula:

(1) $$\begin{array}{c} \text{MNF}=\frac{\int \infty \;0\;\omega P\left(t,\omega \right)\text{d}\omega }{\int \infty \;0\;P\left(t,\omega \right)\text{d}\omega }, \end{array}$$

where (*t*) is equal to the power spectrum of EMG signals based on wavelet packet transformation.

The normalised processing equation of the data obtained from each participant within each 3-second epoch is as follows:

(2) $$\begin{array}{c} x_{\text{Normalized}}=\frac{x_{i}-\;x_{\min}}{x_{\max}-x_{\min}}, \end{array}$$

where *x*_Normalized_ is equal to the normalised value of raw data *x*_*i*_ and *x*_max_ and *x*_min_ indicate the maximum and minimum values of series *X*, respectively.

### 2.5. Grey Relational Grade Calculation

The EMG MNFs of six muscle groups were selected as inspection sequences to choose power or cadence as the standard sequence. The normalisation of each standard and inspection sequence data were calculated by dividing the average value of the sequence. We then calculated the grey relational coefficient using the preprocessed sequences and Deng's formula for grey relational grade. The formula is shown as follows:

(3) $$\begin{array}{c} \text{corr}\left(x0\left(k\right),\;xi\left(k\right)\right)=\frac{\Delta \min+p\Delta \max}{\Delta 0i\left(k\right)+p\Delta \max}, \end{array}$$

where *i* = 1, 2, 3,…, *m* and *k* = 1, 2, 3,…, *n*; x0 and xi indicate the standard sequence and inspected sequence, respectively. Δ0i = ||*x*0(*k*) − *xi*(*k*)|| is the diﬀerence between *x*0 and *xi*. Δmin = ∀imin.min. ∀k||*x*0(*k*) − *xi*(*k*)|| and Δmax = ∀imax.max. ∀k||*x*0(*k*) − *xi*(*k*)||. *p* is the distinguishing coefficient and *p*∈[0,1]. According to previous research, we used *p* = 0.5 in this study.

To calculate the grey correlation coefficient, its mean value is taken as the grey correlation grade (CORR), as determined by the following equation:

(4) $$\begin{array}{c} \text{CORR}\left(x0,\;xi\right)=\frac{1}{n}\sum_{k=1}^{n}\text{corr}\left(x0\left(k\right),xi\left(k\right)\right). \end{array}$$

In this study, the grey relational grade of CORR ranged from 0 to 1. A higher CORR value indicates that the trend of change between the EMG index and power or cadence is closer, and thus, more significantly affects exercise performance.

MATLAB R2016 software (MathWorks, Natick, MA, USA) was used for data processing.

### 2.6. Statistical Analysis

Normality distribution of data was assessed using Kolmogorov–Smirnov test, and one-way repeated-measures analysis of variance (ANOVA) was used to determine differences between pedalling performance (power or cadence) and EMG index in every 3-second epoch. The Spearman rank cross-correlation analysis was used to observe any correlations between dependent variables, namely, power, cadence, and EMG MNF, and all-out cycling exercise duration time. The Pearson cross-correlation analysis was used to identify correlations between power, cadence, and MNF and demographic information (age and BMI). The nonparametric Mann–Whitney *U* test was used to compare differences between power, cadence, and EMG MNF at each phase point between male and female participants. Repeated-measures ANOVA was used to compare the grey relational grades of different EMG indices and pedalling performance (power and cadence). Statistical analyses were performed using SPSS for Windows version 13.0 (SPSS Inc., Chicago, IL, USA). All significant thresholds were fixed at *α* = 0.05. Data were reported as mean ± standard deviation (SD).

## 3. Results

The average power output and cadence of all participants calculated for every 3-second period over the exercise duration are presented in Figure 3. From the 3^rd^ pedalling epoch, the power and cadence showed a gradual, approximately linear downward trend. Spearman cross-correlation analysis revealed that exercise performance (power and cadence) decreased significantly with increasing duration time (power: *ρ* = −0.845, *P* ≤ 0.001; cadence: *ρ* = −0.783, *P* ≤ 0.001). Based on one-way repeated-measures ANOVA, we found statistically significant differences in power and cadence between the 2^nd^ and 10^th^ pedalling epochs (power: *F* = 33.421, *P* ≤ 0.001; cadence: *F* = 45.030, *P* ≤ 0.001).

Moreover, Pearson cross-correlation analysis revealed that both age and BMI had no significant influence on power and cadence (all *P* > 0.05). Similarly, the Mann–Whitney *U* test revealed no significant differences between power and cadence at each phase point (normalised value) between male and female participants (all *P* > 0.05).

Figure 4 displays the EMG MNF of each muscle calculated for every 3-second period during a 30-second all-out pedalling exercise. The MNF of RF, VAS, TA, and GAS was significantly influenced by the duration time (RF : *F* = 9.288, *P* ≤ 0.001; VAS : *F* = 5.460, *P* ≤ 0.01; TA : *F* = 11.579, *P* ≤ 0.001; and GAS : *F* = 12.227, *P* ≤ 0.001), whereas no evidence of an association was found between the duration time and the MNF of HAM and SOL (HAM : *F* = 1.821, *P* > 0.05; SOL : *F* = 1.214, *P* > 0.05). In addition, Spearman cross-correlation analysis revealed significantly negative correlations between the duration time and the MNF of each muscle (RF: *ρ* = −0.589, *P* ≤ 0.001; VAS: *ρ* = −0.519, *P* ≤ 0.001; HAM: *ρ* = −0.329, *P* ≤ 0.05; TA: *ρ* = −0.687, *P* ≤ 0.001; GAS: *ρ* = −0.686, *P* ≤ 0.001; and SOL: *ρ* = −0.341, *P* ≤ 0.05).

Moreover, based on Pearson cross-correlation analysis, we found that neither age nor BMI had a significant influence on the MNF of each muscle (all *P* > 0.05). We also found using the Mann–Whitney *U* test no significant differences between the MNF of each muscle at each phase point and male and female participants (all *P* > 0.05).

Table 1 shows the grey relational grade of the EMG indices and pedalling performance. We determined that different muscles had significantly different grey relational grade values (*F* = 11.793, *P* ≤ 0.001). Further, there was no significant main effect of performance indices (*F* = 0.722, *P* > 0.05), but a significant interaction effect between EMG and performance indices was found (*F* = 1.006, *P* > 0.05). Multicomparison results revealed that the grey relational grade of TA was higher than other muscles (*P* < 0.05), whereas the grey relational grades of HAM and SOL were significantly lower than other muscles (*P* < 0.05).

## 4. Discussion

The main finding of our study was that the EMG MNF of TA had the highest grey relational grades of exercise performance among all six measured muscle groups; in contrast, the grey relational grades of HAM and SOL were significantly lower than the other muscles. To our knowledge, this study is the first to explore the relationship between exercise performance decline and the fatigue degree of each lower limb muscle during 30-second all-out sprint cycling.

In this study, each participant performed a strenuous all-out sprint cycling exercise, during which most lower limb muscles contracted at very high forces and tended to fatigue quickly. As a result, the EMG MNF of RF, VAS, TA, and GAS decreased significantly during the entire exercise process, indicating that the fatigue of these muscles developed quickly and continuously during the entire exercise process. Correspondingly, we found that exercise capacity and performance (power and cadence) showed a significant decline from the 3^rd^ 3-second epoch and developed progressively during the latter epochs.

We also determined that the grey relational grade of TA was higher than that of other muscles, indicating a closer relationship between TA fatigue and total exercise performance decline during 30-second all-out sprint cycling. This finding is consistent with that of Martin and Brown, who reported an up to 63% decrease in ankle joint power during a 30-second cycling sprint [18]. During 30-second sprint cycling in our cohort, the EMG MNF of TA showed a steady and nearly linear decrease, indicating a significant and severe fatigue development of the TA muscle. It has been suggested that TA plays a significant role in the directional control of force production on the pedal, and thus influences cycling technique and pedalling effectiveness [19, 20]. The significant impact of TA fatigue on exercise performance decline during this cycling exercise in our cohort is in agreement with these previous findings.

Previous studies have reported a close relationship between exercise performance decline and muscle fatigue of VAS, RF, and GAS during short-time sprint cycling exercise. Furthermore, it was proposed that VAS and GAS play a key role in the total power contribution during maximal sprint cycling, whereas RF was an important muscle in energy transfer between joints at critical times [21]. RF was also found to be more susceptible to fatigue development than other quadriceps femoris muscles during sprint cycling exercise due to greater activation of muscle fibres as well as the high composition of type II muscle fibres [22–24]. In this study, the average grey relational grades between exercise performance and VAS, RF, and GAS were all greater than 0.74 and significantly higher than the grey relational grades of HAM and SOL, indicating a close relationship between exercise performance decline and muscle fatigue of VAS, RF, and GAS during 30-second all-out cycling.

Regarding the muscles of HAM and SOL, previous studies have found no significant roles for these muscles in force production, power transfer, and fatigue development during continuous sprint cycling, which were consistent with the results of the present study [3, 20, 25]. We found no significant interaction influence of duration time on the MNFs of HAM and SOL, a finding which may be explained by their lower activation level and high composition of type I muscle fibres [3, 20, 25]. It has been suggested that approximately ∼80–85% of the power produced over a pedal cycle is generated during leg extension (i.e., the downstroke), whilst ∼15–20% is produced during leg flexion (i.e. the upstroke) [26], which may also explain the significant roles of TA, RF, and VAS during sprint cycling. In a broader context, these findings indicate that the anaerobic endurance training of HAM and SOL for improving 30-second all-out sprint cycling exercise performance and the whole anaerobic endurance ability of lower limb muscles is less of a concern as the two muscles are not apt to fatigue during exercise.

A few limitations should be acknowledged in the current study. Firstly, the number of male and female participants in our cohort is distinct, which may affect the universality and reliability of the results [27–29]. Addressing this potential issue, we evaluated the power, cadence, and MNF for each muscle in our cohort, and our data demonstrated similar changes in the indices and metrics between male and female participants. In fact, there were no significant differences between male and female participants, thereby excluding potential sex-specific differences in the results. Additionally, our original power analysis indicated eight participants were statistically needed for our study, but we recruited ten. Secondly, we examined the EMG activities of eight leg muscles, and several muscles, including the gluteus maximus (GMax) and medial GAS (GAS_M_), were not considered. According to a previous study, the absence of GAS_M_ data is not critical as the function of GAS_M_ can be inferred by the activity of the lateral GAS [21]. However, the functional role of GMax cannot be replaced by other muscles, so the absence of GMax is a limitation of the current study. Lastly, except for the main effect of fatigue of each lower limb muscle on the decline of exercise performance, changes of muscle coordination induced by fatigue may also influence exercise performance during 30-second all-out sprint cycling [3], a possible effect which was not considered in our study. Nevertheless, despite these limitations, our current findings provide insights towards understanding the relationship between the fatigue of lower limb muscles and exercise performance during a 30-second all-out cycling exercise.

## 5. Conclusion

In conclusion, RF, VAS, GAS, and TA progressively tired during a 30-second all-out sprint cycling exercise. Of the muscles evaluated, the degree of fatigue of TA showed the greatest association with exercise performance decline, whereas the muscle fatigue of RF, VAS, and GAS also significantly impacted exercise performance during a 30-second all-out sprint cycling exercise. The findings may provide insights for coaches and cyclists to better understand the physiology and changes related to high-impact exercise and aid the design of more effective training programmes.

## Figures and Tables

**Figure 1:** Experimental protocol.

**Figure 2:** Electromyogram electrode locations of each tested muscle.

**Figure 3:** The average power and cadence of all 10 participants calculated for every 3-second period during a 30-second all-out cycling exercise.

**Figure 4:** The EMG MNF of each muscle calculated for every 3-second period during a 30-second all-out cycling exercise. (a) RF, (b) VAS, (c) HAM, (d) TA, (e) GAS, and (f) SOL. An ^*∗*^indicates a significant main effect of sprint duration time on EMG MNF, whereas # indicates a significant negative correlation between the EMG MNF and sprint duration time.

**Table 1:** Grey relational grades between pedalling performance and the EMG MNF of each.

	RF	VAS	HAM	TA	GAS	SOL
Power	0.77 ± 0.13	0.74 ± 0.17	0.68 ± 0.17^▼^	0.82 ± 0.13^▲^	0.81 ± 0.14	0.67 ± 0.16^▼^
Cadence	0.83 ± 0.11	0.78 ± 0.14	0.67 ± 0.16^▼^	0.93 ± 0.04^▲^	0.81 ± 0.06	0.68 ± 0.17^▼^

*Note.* ▲ and ▼, respectively, indicate significantly higher and lower grey relational grade values than other muscles.

## Data Availability

The data used to support the findings of this study are available from the corresponding author upon request.
